# Gastrodin relieves inflammation injury induced by lipopolysaccharides in MRC‐5 cells by up‐regulation of miR‐103

**DOI:** 10.1111/jcmm.14826

**Published:** 2019-11-25

**Authors:** Zhuona Xi, Yahong Qiao, Jifang Wang, Hongjian Su, Zhen Bao, Hongyan Li, Xiaoming Liao, Xiaolan Zhong

**Affiliations:** ^1^ Department of Respiration Ward II Henan Provincial Chest Hospital Zhengzhou China; ^2^ Department of Internal Medicine Huadu District People's Hospital of Guangzhou Guangzhou China; ^3^ Department of Integrated Chinese and Western Internal Medicine Huadu District People's Hospital of Guangzhou Guangzhou China; ^4^ Department of Quality Control Huadu District People's Hospital of Guangzhou Guangzhou China

**Keywords:** apoptosis, chronic obstructive pulmonary disease (COPD), NF‐κB, p38/JNK

## Abstract

The beneficial function of gastrodin towards many inflammatory diseases has been identified. This study designed to see the influence of gastrodin in a cell model of chronic obstructive pulmonary disease (COPD). MRC‐5 cells were treated by LPS, before which gastrodin was administrated. The effects of gastrodin were evaluated by conducting CCK‐8, FITC‐PI double staining, Western blot, qRT‐PCR and ELISA. Besides this, the downstream effector and signalling were studied to decode how gastrodin exerted its function. And dual‐luciferase assay was used to detect the targeting link between miR‐103 and lipoprotein receptor‐related protein 1 (LRP1). LPS induced apoptosis and the release of MCP‐1, IL‐6 and TNF‐α in MRC‐5 cells. Pre‐treating MRC‐5 cells with gastrodin attenuated LPS‐induced cell damage. Meanwhile, p38/JNK and NF‐κB pathways induced by LPS were repressed by gastrodin. miR‐103 expression was elevated by gastrodin. Further, the protective functions of gastrodin were attenuated by miR‐103 silencing. And LRP1 was a target of miR‐103 and negatively regulated by miR‐103. The in vitro data illustrated the protective function of gastrodin in LPS‐injured MRC‐5 cells. Gastrodin exerted its function possibly by up‐regulating miR‐103 and modulating p38/JNK and NF‐κB pathways.

## 1 INTRODUCTION

Chronic obstructive pulmonary disease (COPD) is a complex systemic disorder characterized by both local pulmonary inflammation and systemic inflammation.^1^ This disease mainly manifests by chronic and progressive cough, sputum production and dyspnoea after exercise^2^ which significantly affects the quality of life and exercise endurance of patients.^3^ Until now, no reliable information suggests that the present pharmacotherapy of modern medicine can reverse the progressive decline of pulmonary function in the natural course of COPD.^4^ So, preventing COPD is one of the major options of management of this illness.

*Gastrodia eleta* is one of the traditional Chinese herbal medicines that is used in ancient time to treat many diseases, including migraines, dizziness, tetanus, epilepsy, infantile convulsions, rheumatism and numbness of the limbs. Gastrodin (4‐hydroxybenzyl alcohol 4‐O‐beta‐d‐glucopyranoside) is a major active constituent of *Gastrodia eleta*. Recent decades, various pharmacological functions of gastrodin have been reported, including anti‐apoptosis, anti‐inflammation, antioxidant activity, lipid regulation^5^, ^6^ and so forth. Thereby, gastrodin has been considered as a potential therapeutic agent for diverse diseases such as Tourette syndrome,^7^ myocardial infarction,^8^ alcoholic liver disease^6^, ^9^ and acute lung injury.^10^ However, the effects of gastrodin on COPD were not studied previously.

microRNAs (miRNAs) are a sort of small non‐coding RNAs that are latterly discovered. They constitute approximately 1% of the total coding genes, and regulate more than 1/3 of protein‐coding genes post‐transcriptionally, which form the largest molecule regulation network. Because of this, miRNAs can participate in various physiological and pathological processes, including the onset and development of COPD.^11^, ^12^, ^13^ For instance, in vivo and in vitro data demonstrated that miR‐3202 could protect smokers from COPD.^14^ Likewise, miR‐181c was able to inhibit COPD which was induced by smoke.^15^ In COPD, miR‐103 was reported to be one of the aberrantly expressed miRNAs.^16^ Besides that, miR‐103 could participate in the regulation of inflammation in many aspects of human body, such as vasculature,^17^ adipose tissue^18^ and epicardial adipose tissue.^19^ However, the functional impacts of miR‐103 in COPD have not been studied before.

This study attempted to investigate the effect of gastrodin on a cell model of COPD, which was constructed by stimulating human lung fibroblast MRC‐5 cells with lipopolysaccharides (LPSs). The expression change in miR‐103 was also studied to decode the mechanism of which gastrodin exerted its function.

## 2 MATERIALS AND METHODS

### 2.1 Cell treatment

MRC‐5 cells (ATCC) were cultured in EMEM (ATCC) which supplemented with 10% foetal bovine serum (Gibco). The cells were subcultured in 75‐cm^2^ flask and maintained at 37°C in humidified atmosphere with 5% CO_2_.

Cells were treated by 10 μg/mL LPS (Sigma‐Aldrich) for 6 hours as described elsewhere.^20^

Gastrodin (≥98% (HPLC), Sigma‐Aldrich) was dissolved in DMSO (Sigma‐Aldrich) to make a storage solution. Before use, the solution was diluted with EMEM to final concentrations of 50‐300 μg/mL. The cells were treated by gastrodin for 24 hours before LPS stimulation.

### 2.2 Transfection

miR‐103 mimic, miR‐103 inhibitor (anti–miR‐103) and the negative control (NC) were synthesized by GenePharma. Before transfection, cells were seeded into 6‐well plates at the density of 5 × 10^5^/well. Cells were transfected with a final concentration of 5 nmol/L for miRNA mimic and 50 nmol/L for miRNA inhibitor through Lipofectamine 3000 (Invitrogen) following the producer's instructions. Transfection complexes were formed as follows: 100 pmoles miR‐103–related sequences and 5 μL lipofectamine 3000 were blended, respectively, with 125 μL Opti‐MEM (Invitrogen), keeping them in the room for 10 minutes under serum‐free conditions. Cells were washed twice with PBS, and relative transfection complexes were put into every well. After 48 hours, the stably transfected cells were chosen for about 4 weeks through the culture medium with 0.5 mg/mL G418 (Sigma‐Aldrich). G418‐resistant cells were directly gathered latter.

### 2.3 Cell viability

5000 cells in 96‐well plates were treated as indicated. Cell viability was tested by adding 20 μL CCK‐8 solution (Sangon Biotech). 4 hours later, the optical density (OD) at 450 nm was analysed by a microplate reader (Bio‐Rad).

### 2.4 Apoptosis

5 × 10^5^ cells in 6‐well plates were treated as indicated, after which 1 × 10^5^ cells of each sample were stained by using Annexin V‐FITC Apoptosis Detection Kit (Yeasen). FACS can (Beckman Coulter) was utilized to analyse apoptosis rate.

### 2.5 ELISA

Cells in 6‐well plates were treated as indicated, and thereafter, the culture supernatant was collected. Concentrations of MCP‐1, IL‐6 and TNF‐α were tested by ELISA Kits purchased from Abcam.

### 2.6 qRT‐PCR

Cells in 6‐well plates were treated as indicated. RNA extraction was done by using TRIzol (Invitrogen), and the purity was verified by testing the OD values at 260 and 280 nm. To analyse MCP‐1, IL‐6 and TNF‐α levels, PrimeScript™ RT Master Mix and TB Green Fast qPCR Mix (Takara) were utilized and β‐actin acted as an internal control. To analyse the expression of miR‐103, Mir‐X™ miRNA First‐Strand Synthesis Kit and Mir‐X™ miRNA qRT‐PCR TB Green™ Kit (Takara) were utilized and U6 acted as reference controls.

### 2.7 Western blot

The proteins in the pre‐treated cells were isolated by using RIPA buffer (Beyotime). The proteins was separated and probed by the primary antibodies, including anti–Bcl‐2 (sc‐509), anti‐Bax (sc‐20067), anti–cleaved Caspase 3 (sc‐373730), anti–cleaved PARP (sc‐56196), anti–MCP‐1 (sc‐130328), anti–IL‐6 (sc‐57315), anti–TNF‐α (sc‐52746), anti‐p38 (sc‐136210), anti–p‐p38 (sc‐7973), anti–c‐Jun (sc‐376488), anti–p‐c‐Jun (sc‐53182), anti‐JNK (sc‐136533), anti–p‐JNK (sc‐293137), anti‐p65 (sc‐514451), anti–p‐p65 (sc‐136548) and anti–β‐actin (sc‐517582, Santa Cruz Biotechnology). Followed by incubation with the secondary antibodies, the positive bands were developed by BeyoECL Star Kit (Beyotime).

### 2.8 Dual‐luciferase assays

3′‐UTR of lipoprotein receptor–related protein 1 (LRP1) was amplified through PCR and inserted into pmiR‐Report vector (Promega), indicating LRP1 wild type (WT). GeneTailor Site‐Directed Mutagenesis System (Invitrogen) was employed to get LRP1‐mutated type (MUT), which was amplified via PCR and inserted into the same vector. The vectors were cotransfected with miR‐103 mimic and its related control into cells. Dual‐luciferase experiment system (Promega) was employed to get results.

### 2.9 Statistics

Data presented as mean ± SD. Statistical difference was tested by SPSS 19.0 software (Chicago, IL) and presented as asterisk. Student's *t* test and ANOVA with Tukey post hoc analysis were conducted to compare the significant difference. *P* < .05 was considered as significant difference.

## 3 RESULTS

### 3.1 LPS injured MRC‐5 cells

MRC‐5 cells were stimulated by 10 μg/mL LPS for 6 hours. As expected, cell viability was repressed (*P* < .05, Figure 1A), whereas apoptosis rate was increased (*P* < .05, Figure 1B) by LPS. These phenomena were accompanied by the down‐regulation of Bcl‐2, the up‐regulation of Bax and the cleavage of Caspase 3 and PARP (all *P* < .05, Figure 1C,D). Meanwhile, the expression and release of MCP‐1, IL‐6 and TNF‐α in MRC‐5 cells were promoted by LPS (all *P* < .05, Figure 1E‐G). All these demonstrated the inflammatory injury in MRC‐5 cells induced by LPS.

**Figure 1:** LPS injured MRC‐5 cells. MRC‐5 cells were stimulated by 10 μg/mL LPS for 6 h. (A) Viability, (B) apoptosis rate, (C‐D) apoptosis‐related proteins' expression, and (E) mRNA level, (F) protein level and (G) release of MCP‐1, IL‐6 and TNF‐α were analysed by CCK‐8, FITC‐PI double staining, Western blot, qRT‐PCR and ELISA. * indicates *P* < .05, n = 3

### 3.2 Gastrodin prevents LPS‐induced injury in MRC‐5 cells

Various concentrations of gastrodin were utilized to treat MRC‐5 cells for 24 hours. As result shown in Figure 2A, no significant changes were observed in cell viability, indicating gastrodin with concentrations ranged from 50 to 300 μg/mL had no cytotoxicity. However, gastrodin could significantly increase cell viability in LPS‐induced cells in a dose‐dependent way (*P* < .05, Figure 2B). As 200 μg/mL gastrodin led to the highest viability in LPS‐induced cells, it was selected as an optimum concentration used in the following. We found that pre‐treating MRC‐5 cells with gastrodin attenuated LPS‐induced apoptosis, as apoptosis rate was decreased (*P* < .05, Figure 2C), Bcl‐2 was up‐regulated, Bax was down‐regulated, and the cleavage of Caspase 3 and PARP was repressed (all *P* < .05, Figure 2D,E). Not surprisingly, the expression and release induced by LPS were attenuated when pre‐treating with gastrodin (all *P* < .05, Figure 2F‐H).

**Figure 2:** Gastrodin prevents LPS‐induced injury in MRC‐5 cells. (A) The viability of MRC‐5 cells was analysed by CCK‐8, following by administration with various concentrations of gastrodin for 24 h. (B) MRC‐5 cell viability was analysed after treating with the indicated concentration of gastrodin for 24 h and then LPS. MRC‐5 cells were treated by 200 μg/mL gastrodin for 24 h and then LPS. (C) Apoptosis rate, (D‐E) apoptosis‐related proteins' expression, and (F) mRNA level, (G) protein level and (H) release of MCP‐1, IL‐6 and TNF‐α were analysed by FITC‐PI double staining, Western blot, qRT‐PCR and ELISA. * indicates *P* < .05, n = 3

### 3.3 Gastrodin inhibits p38/JNK and NF‐κB pathways

The effects of gastrodin on p38/JNK and NF‐κB pathways were investigated. As seen in Figure 3A‐D, phosphorylation of p38, c‐Jun, JNK and NF‐κB p65 was significantly induced by LPS (all *P* < .05). However, pre‐treatment of gastrodin ameliorated the phosphorylation induced by LPS (*P* < .05). It seems that gastrodin could impede the inductive impacts of LPS on p38/JNK and NF‐κB pathways.

**Figure 3:** Gastrodin inhibits p38/JNK and NF‐κB pathways. MRC‐5 cells were treated by 200 μg/mL gastrodin for 24 h and 10 μg/mL LPS for 6 h. Expression of (A‐B) p38, Jun and JNK, and (C‐D) NF‐κB p65 was analysed by Western blot. * indicates *P* < .05, n = 3

### 3.4 Gastrodin up‐regulates miR‐103 expression

Next, miR‐103 expression was analysed following LPS and gastrodin treatment. Data in Figure 4 displayed that miR‐103 was low expressed in LPS‐induced cell (*P* < .05), whereas was highly expressed in gastrodin‐treated cell even under LPS conditions (*P* < .05).

**Figure 4:** Gastrodin up‐regulates miR‐103 expression. MRC‐5 cells were treated by gastrodin plus LPS. miR‐103 expression was analysed by qRT‐PCR. * indicates *P* < .05, n = 3

### 3.5 Gastrodin prevents LPS‐induced injury via miR‐103

Finally, miR‐103 expression in MRC‐5 cells was silenced by transfection to decode the importance of miR‐103 in gastrodin's protective action. Data in Figure 5A displayed the significant down‐regulation of miR‐103 by transfection with specific inhibitor (*P* < .05), indicating miR‐103 expression in MRC‐5 cells was successfully silenced. Post‐transfection, cells were treated by gastrodin and then LPS. Results in Figure 5B‐E showed that gastrodin's effect on MRC‐5 cells viability and apoptosis were flattened when miR‐103 was silenced (*P* < .05). Also, gastrodin did not repress LPS‐induced release of pro‐inflammatory cytokines when miR‐103 was silenced (*P* < .05, Figure 5F‐H).

**Figure 5:** Gastrodin prevents LPS‐induced injury via miR‐103. (A) miR‐103 expression was analysed by qRT‐PCR, after MRC‐5 cells were transfected with miR‐103 inhibitor (anti–miR‐103) or the negative control (NC). The transfected cells were treated by gastrodin plus LPS. (B) Viability, (C) apoptosis rate, (D‐E) apoptosis‐related proteins' expression, and (F) mRNA level, (G) protein level and (H) release of MCP‐1, IL‐6 and TNF‐α were analysed by CCK‐8, FITC‐PI double staining, Western blot, qRT‐PCR and ELISA. * indicates *P* < .05, n = 3

### 3.6 LRP1 was a target of miR‐103

To investigate the target of miR‐103, TargetScan (http://www.targetscan.org) and microRNA database (http://www.microrna.org) were employed to predict the binding site between LRP1 and miR‐103 (Figure 6A). Besides, the overexpression of miR‐103 was achieved through transfection with miR‐103 mimic (*P* < .001, Figure 6B). And Figure 6C,D revealed that the mRNA and protein levels of LRP1 were notably reduced by miR‐103 overexpression (*P* < .05), while were notably increased by the inhibition of miR‐103 (*P* < .01). Meanwhile, dual‐luciferase assay revealed that luciferase activity of miR‐103 mimic + LRP1‐WT group was greatly reduced (*P* < .05), whereas that of miR‐103 mimic + LRP1‐MUT group was no changed (Figure 6E). Thus, LRP1 was a target gene of miR‐103 and was down‐regulated by miR‐103.

**Figure 6:** LRP1 was a target of miR‐103. (A) The binding site of miR‐103 and LRP1 was analysed through TargetScan and microRNA database. (B) Expression of miR‐103 was examined through qRT‐PCR after transfection with miR‐103 mimic. Expression of LRP1 was examined through qRT‐PCR (C) and Western blot (D) after transfection with miR‐103 mimic and anti–miR‐103. (E) The target relationship between miR‐103 and LRP1 was examined by dual‐luciferase reporter assay. * indicates *P* < .05, ** indicates *P* < .01 and *** indicates *P* < .001, n = 3

## 4 DISCUSSION

Considering COPD is a progressive disease, the damaged pulmonary function is hard to be reversed. Thus, preventing COPD has become a promising method for COPD management and a small fraction of researches have focused on the beneficial effects of traditional Chinese herbal medicine on this disease.^21^ This study attempted to investigate the potential of gastrodin for COPD management. To this end, LPS was applied to treat MRC‐5 cells to construct a cell model of COPD. Much was known that LPS is effective in inducing inflammatory response.^22^, ^23^ This phenomenon was also appended in this study that LPS induced apoptosis and the release of MCP‐1, IL‐6 and TNF‐α in MRC‐5 cells. Interestingly, pre‐treating MRC‐5 cells with gastrodin attenuated LPS‐induced apoptosis and pro‐inflammatory cytokines release. Further studies found that gastrodin exerted protective functions possibly be associated with the up‐regulated miR‐103 expression and the inhibited p38/JNK and NF‐κB pathways.

Despite the functional effects of gastrodin on COPD are unstudied before, its effects on other types of inflammatory diseases have been previously reported. For the selected examples, gastrodin is capable of relieving chronic inflammatory pain^24^ and neuroinflammation.^25^ gastrodin may even attenuate LPS‐induced acute lung injury.^10^ Thus, it seems rationality that gastrodin could also protect MRC‐5 cells against LPS‐induced inflammatory injury. Besides that, gastrodin is reported to be an effective agent in resisting apoptosis made by various stimulations, such as hypoxic ischaemia,^26^ ethanol,^9^ high glucose^27^ and LPS.^28^ Consistently, gastrodin exhibited anti‐apoptosis effect in our experimental system. Moreover, gastrodin prevented MRC‐5 cell apoptosis possibly via a mitochondrial‐dependent way, as the expression of main regulators Bcl‐2 and Bax of this process was altered.

Much was known about the inductive impacts of LPS on various signalling pathways, such as JNK, NF‐κB and p38MAPK.^29^ These three pathways can be activated under cigarette stimulation, which can induce inflammatory response and drive the initiation of COPD.^30^, ^31^, ^32^ Thus, inhibition of p38/JNK and NF‐κB pathways has been considered as effective strategy for treating COPD. Herein, gastrodin was found to be effective in inhibiting LPS‐induced p38/JNK and NF‐κB pathways, which were in line with the findings reported elsewhere.^33^, ^34^ The results indicated that gastrodin prevented LPS‐induced injury in MRC‐5 cells through these two signalling.

Despite the underlying mechanisms of which herbal medicines exert their beneficial function are still unclear, scientists believed that miRNAs are main targets of them.^35^ In regard to gastrodin, less was known about its regulation on miRNA expression. To date, only one report demonstrated that gastrodin could protect cardiomyocytes through up‐regulating miR‐21.^8^ In the current study, we for the first time illustrated that gastrodin could elevate miR‐103 expression. And the protective effects of gastrodin towards MRC‐5 cells were partially flattened by miR‐103 silence. Altogether, gastrodin prevented LPS‐induced injury in MRC‐5 cells possibly by up‐regulating miR‐103. Additionally, miR‐103's expression was reported to be low in hypoxic pulmonary hypertension.^36^ Besides, it was proved to promote LPS‐induced inflammatory damage in HK‐2 cells.^37^ However, other studies found that miR‐103 reduced apoptosis in LPS‐caused PC12 cell injury to play protective roles.^38^ This contradiction may due to the different cell lines or different irritations used in experimental system. In the future, it will be interesting to explore the functional mechanism of miR‐103 in different cell situations.

Further, LRP1, a member of LDLR superfamily,^39^ was reported to be a modulator of the inflammatory response in lung.^40^ It controls the recruitment of inflammatory lung cells and triggers pulmonary inflammation. Leslie et al^41^ found that the up‐regulation of miR‐103 mediated by p53 could lead to the suppression of LRP1 translation and cell death. Consistently, our study also found that anti–miR‐103's transfection raised apoptosis in LPS and gastrodin‐treated MRC‐5 cells, indicating that apoptosis was reduced by miR‐103. Besides, it is worth noting that LRP1 was a target of miR‐103 and was down‐regulated by miR‐103. This finding demonstrated the molecular mechanism downstream to the gastrodin ‐induced miR‐103 up‐regulation. Further work is needed to explore whether miR‐103 participates in anti‐inflammatory effects of gastrodin by regulating LRP1.

To conclude, we offered a new feasible molecular explanation of gastrodin in protecting MRC‐5 cells from LPS‐caused damage. The in vitro data illustrated that the apoptosis and pro‐inflammatory cytokines release were repressed by gastrodin. Moreover, gastrodin exerted its function possibly via up‐regulating miR‐103 and inhibiting p38/JNK and NF‐κB pathways. Our findings suggested that the beneficial effects of gastrodin may be developed as a new therapeutic approach in the treatment of COPD. Actually, gastrodin used as a traditional Chinese herbal medicine for many years, and this is the first report of studying the effects of gastrodin on COPD. It has important clinical significance for the treatment of COPD. More efforts, especially in vivo experiments, are required to further define gastrodin's effect in COPD.

## CONFLICT OF INTEREST

The authors declare that they have no competing interests.

## AUTHORS' CONTRIBUTIONS

Zhuona Xi, Xiaoming Liao and Xiaolan Zhong conceived and designed the experiments. Yahong Qiao, Jifang Wang, Hongjian Su, Zhen Bao and Hongyan Li performed the experiments and analysed the data. Zhuona Xi, Xiaoming Liao and Xiaolan Zhong wrote the manuscript.

## Data Availability

The data sets used and/or analysed during the current study are available from the corresponding author on reasonable request.
